# A Multi-Thresholding-Based Discriminative Neural Classifier for Detection of Retinoblastoma Using CNN Models

This article has been retracted.

**DOI:** 10.1155/2023/5803661

**Published:** 2023-02-06

**Authors:** Parmod Kumar, D. Suganthi, K. Valarmathi, Mahendra Pratap Swain, Piyush Vashistha, Dharam Buddhi, Emmanuel Sey

**Affiliations:** ^1^Department of Electronics and Information Engineering, Jiangxi University of Engineering, Xinyu City, Jiangxi, China; ^2^Department of Computer Science, Saveetha College of Liberal Arts and Sciences, SIMATS, Chennai, India; ^3^Department of Computer Science and Engineering, Panimalar Engineering College, Chennai, India; ^4^Department of Pharmaceutical Sciences and Technology, Birla Institute of Technology, Mesra, Ranchi, India; ^5^Department of Computer Engineering & Applications, GLA University, Mathura, Uttar Pradesh, India; ^6^Division of Research & Innovation, Uttaranchal University, Dehradun, Uttarakhand, India; ^7^Kwame Nkrumah University of Science and Technology, Kumasi, Ghana

## Abstract

Cancer is one of the vital diseases which lead to the uncontrollable growth of the cell, and it affects the body tissue. A type of cancer that affects the children below five years and adults in a rare case is called retinoblastoma. It affects the retina in the eye and the surrounding region of eye like the eyelid, and sometimes, it leads to vision loss if it is not diagnosed at the early stage. MRI and CT are widely used scanning procedures to identify the cancerous region in the eye. Current screening methods for cancer region identification needs the clinicians' support to spot the affected regions. Modern healthcare systems develop an easy way to diagnose the disease. Discriminative architectures in deep learning can be viewed as supervised deep learning algorithms which use classification/regression techniques to predict the output. A convolutional neural network (CNN) is a part of the discriminative architecture which helps to process both image and text data. This work suggests the CNN-based classifier which classifies the tumor and nontumor regions in retinoblastoma. The tumor-like region (TLR) in retinoblastoma is identified using the automated thresholding method. After that, ResNet and AlexNet algorithms are used to classify the cancerous region along with classifiers. In addition, the comparison of discriminative algorithm along with its variants is experimented to produce the better image analysis method without the intervention of clinicians. The experimental study reveals that ResNet50 and AlexNet yield better results compared to other learning modules.

## 1. Introduction

Ophthalmology is a branch of medicine, and surgeries that focuses on the diagnosis and treating a wide variety of conditions that affect the eyes are needed. The eye is the organ that takes in light and transmits information about what it sees to the brain, which then forms a picture. Several structures are seen in someone's eyes. The pupil lets light enter the eye. A brilliantly pigmented round muscle, the iris, gives us eye color. A transparent cornea covers the pupil and iris. Together with the crystalline lens, it produces a sharp vision at the retinal receptor level. The globe, the orbit (sometimes known as the eye socket), and the adnexa are the three primary components of the eye. Tumors of the eye can be either benign or malignant. Eye tumors, also known as ocular tumors, can originate in any part of the eye. When healthy cells in or around the eye undergo malignant changes, they begin to multiply uncontrollably and spread to other parts of the body, which ultimately results in the production of malignant cells. Ocular tumors are another name for eye tumors. A mass of cells that develops erratically is called a tumor. It might be malignant or not. Malignant is the medical term for cancerous tumors. Benign tumors are those that are not cancerous. The tissues around the eyeball are impacted by orbital malignancies. The orbit is the name for this. Additionally, the eyeball's moving muscles and its associated nerves may be impacted. The tear ducts and eyelids may also be impacted. Adnexal tumors are cancers that affect these structures. Commonly, benign moles develop into malignant melanomas. A benign tumor will grow in size but will not spread to other organs. Benign tumor cells are noncancerous tumors which cause inflammation around the eye. A malignancy that originates in the eyeball is referred to as an intraocular tumor, which literally means “inside the eye.” Primary intraocular malignancies and secondary intraocular cancers are the two distinct subtypes of intraocular tumors that can manifest in the eye. Primary intraocular cancers start inside the eye. Melanoma is the most common primary eye cancer in adults [1]. Retinoblastoma (RB) is the most common intraocular malignancy in children. Secondary intraocular malignancies originate on the surface of the globe and then spread into its interior. Retinoblastoma is a kind of cancer that seldom affects adults and children under the age of five. If it is not identified at an early stage, it can sometimes result in vision loss. It affects the retina in the eye as well as the area around the eye, such as the eyelid. To locate the malignant spot in the eye, MRI and CT scans are frequently performed. The clinicians' assistance is required for the current cancer region identification screening procedures to identify the affected areas. Modern healthcare systems create a quick method of disease diagnosis. Retinoblasts make up retinoblastoma (basophilic cells with hyperchromatic nuclei and scanty cytoplasm). The majority of retinoblastomas are undifferentiated; however, variable levels of differentiation are evident because rosettes occur. Although they are not technically “eye tumors,” their incidence is much higher than that of primary intraocular malignancies. Malignancies of the breast and lung are the most prevalent primary tumors that can spread to the eye and cause secondary cancers. The uvea is where the vast majority of these malignancies have metastasized and migrated to the eyeball. The thin layer of light-sensitive tissue that covers the back of the eye is called the retina. It is the reason why we are able to see because when a light signal is received by the eye, it is sent to the brain via the retinal nerve fiber layer. Retinoblastoma can affect either one eye or both eyeballs, depending on which eye is initially infected. As a result, the child's eye has the appearance of a cat's eye. Retinoblastoma's genetic abnormality causes immature eye cells. These retinal cancer cells spread. This spread might harm the spine and brain. A biopsy is used to diagnose most malignancies. During a biopsy, the doctor takes a sample of the tumor for microscopic analysis. Due to two factors, biopsies are infrequently utilized to diagnose retinoblastoma. A biopsy from an eye tumor can spread cancerous cells outside the eye and is challenging to perform. Experienced doctors can frequently identify retinoblastoma without doing a biopsy, and it seldom goes undiagnosed in youngsters with other eye conditions. Robots with artificial intelligence mimic human cognition. Any system that uses machine learning is capable of picking up different patterns and characteristics without human interaction. Imaging tests can be used (1) to determine if an eye tumor is retinoblastoma, (2) to determine tumor size and spread, and (3) to evaluate treatment. Image diagnosis of retinoblastoma includes different methods like ultrasound imaging, magnetic resonance imaging (MRI), and computed tomography (CT) scan [2]. The imaging techniques show the position of the retina in the eye, and the photographs also allow clinicians to investigate a patient's retina, diagnose retinal mutations, and analyze retinal findings. Machine learning is a pattern segmentation procedure that includes a learning approach to understand what distinguishes underlying patterns. Deep learning is the fastest-growing machine learning technology. DL simulates human brain functioning using artificial neural networks. Ophthalmology is about to revolutionize eye screening, diagnosis, and treatment. Deep learning technology could alter ophthalmology treatment. Ophthalmology diagnostic tools provide a computerized picture of eye components. Ophthalmology is a good fit for DL algorithms. DL algorithms in ophthalmology will revolutionize ophthalmologists' work. In the coming years, intelligent technology will aid in eye cancer screening and detection. As DL technology advances, it will be further incorporated into ophthalmic care, freeing practitioners from repetitious duties. Ophthalmologists can improve patient care and interactions. The proposed work is about development of discriminative deep learning model for detection of retinoblastoma using convolutional neural network (CNN) variants with automated multithresholding method.

## 2. Related Works

Retinoblastoma seems to be the most common type of cancerous tumor in kids' eyes. It makes up about 2–3% of all cancers in kids. Leukocoria and strabismus are indeed the two most frequent signs of retinoblastoma. Leukocoria is the most typical early indication of retinoblastoma (a cloudy white pupil). The pupil might seem silvery or yellow under strong light. Other indications include the following: eyes that are not aligned properly, squinted eyes, a larger-than-average pupil, and a murky iris (the colored part of the eye) bad vision. An overview of retinoblastoma, its characteristics, prior discoveries, and research is reviewed in relation to this paper. Allam et al. study the comparison of different artificial intelligence (AI) techniques used to detect the retinoblastoma. This study used AI to classify ocular cancers. Most researches used a two-step strategy to classify eye tumor; they are preprocessing to eliminate noise and classifier. Classifiers employ computer vision techniques, artificial neural networks, and machine learning. Back propagation neural network and image processing yield better performance compared to different AI techniques [3]. Anand et al. report the deep learning technique that allows ophthalmologists towards early prediction and diagnosis of retinoblastoma. LPDMF filter can be used for preprocessing, and the preprocessed images are then segmented using the convolutional neural network (CNN). In retinoblastoma, CNN can be utilized to accurately segment the tumor and the ocular anatomy. The preprocessed images are segmented using a convolutional neural network (CNN) with an architecture known as U-Net to separate the foreground tumor cells from the background's segments of retinoblastoma. The network uses data augmentation techniques to increase the number of training samples while using fewer filters. The seven-layer U-Net architecture has a geometrically increasing number of feature maps at each level and concludes that the suggested model is better than supervised learning algorithms, but still, the quality of the output is not compromised; it requires manual screening to verify the predictive model [4]. Henning et al. proposed a CNN method for detecting leukocoria, which is one of the main symptoms to cause retinoblastoma in the eye. Leukocoria can cause damage to the lens (such as a cataract), vitreous (such as a haemorrhage), or retina (such as retinoblastoma). It may be the first sign of a variety of systemic and intraocular disease processes. The symptom of leukocoria is the light-sensing layer in the back of the eye, typically absorbing the majority of light entering the eye through the pupil. The pupil, however, reflects a little portion of light back out. Due of the reflected reddish orange tint, this is referred to as a red reflex. Red eye is a common effect that flash photography can capture. However, in situations with leukocoria, the pupil of one or both eyes may appear white, yellow, or just pale. 832 eye images are collected from affected children and Flickr, and then, the input images are trained using a traditional three-layer CNN; the model reports a minimum accuracy with small amount of dataset [5]. They studied the mutation of retinoblastomic gene in bladder cancer using machine learning algorithms. The study included CTU scans from 18 patients with RB1 mutation and 54 without. A wrapper-based sequencing feature extraction approach and Pearson's correlation analysis were used for feature selection. Models were created using XGBoost, random forest (RF), and KNN [6]. Priya proposed a CNN-based retinoblastoma detection methods with some segmentation techniques of image processing and calculates the regression of tumors using convex polygon and convex area with the accuracy of 87% [7]. Healthcare has been altered by diagnostic health imaging technology, which now enables earlier diagnosis of medical disorders, lessens the need for pointless invasive exploratory procedures, and improves patient outcomes. The MRA can sometimes gather information that CT scans, ultrasounds, or X-rays cannot by using radio wave energy pulses and a magnetic field. MRA exams are frequently used to gather data on the health of blood flow and blood vessel walls in the legs, neck, brain, and kidneys. MRAs are also used by medical professionals to scan blood arteries for calcium deposits, aneurysms, and clots. In rare circumstances, they might ask for a contrast dye to give the images of the blood vessels in the scan more detail. Strijbis et al. proposed a segmentation method for retinoblastoma using Multiview CNN. The dataset includes 23 patients (17 healthy and 27 RB eyes.). The performance of Multiview CNN can be evaluated using *k*-fold cross validation methods, and it concludes that the proposed method gives better results for segmenting the retinoblastomic image [8].

## 3. Proposed Methodology

Retinoblastoma is perhaps the most frequent pediatric ocular malignancy. In developed countries, retinoblastoma survival rates are 90–99% with current medical treatment. To obtain these survival percentages, retinoblastoma patients must be often evaluated under anesthesia before age 5 for early discovery of new or recurrent tumors, as well as medication and diagnosis of complications. Unlike retinoblastoma, retinoma does not grow or diminish over time. Fundus and OCT images (Figure 1) are used to record the condition of the inner surface of the retina, with the goal of recording the presence of abnormalities and tracking how they evolve over time. OCT is not an eye examination. An eye examination examines eyesight and vision. An OCT scan helps an optometrist to look deeper inside the eyes and their structures than digital retinal imaging. An OCT scan helps an ophthalmologist to assess individual eyesight. A fundus camera, also known as a retinal camera, is a specialized type of low-power microscope that has a camera mounted to it. Its purpose is to take photographs of the internal surface of the eye, such as the retinal, retinal vasculature, optic nerves, macular, and posterior pole [9]. In this study, an image processing approach to classify the cancerous and noncancerous regions in eye images by utilizing Otsu cluster and automated multithresholding was proposed. For accurate categorization, a good image processing approach might be manually chosen. This region selection method can become laborious with more photographs.

A system that analyzes photos and finds suitable places may be more useful. To facilitate image categorization, an appropriate image processing approach is proposed. Segmentation is an essential stage in fundus and OCT image processing. Image segmentation divides an image into distinct sections. Utilizing the properties of a picture's pixels, similarity can be assessed. Segmentation is a pixel categorization method that divides an image into sections with similar content. There are three types of image segmentation: methods for object boundaries based on edges. Closed object regions were created using pixel-based categorization, which uses techniques built from image histogram statistics and region-based approach where regions are created by rapidly evaluating pixels in a region-growing process. To obtain the best threshold value, background removal is the first step. We use an automatic multithresholding at this point to take both dark and light photos of the eye to spot any tumor-like tissue. In the process of processing OCT and fundus images, segmentation is a crucial step. The initial step is background removal in order to get an optimal threshold value. At this stage, use an automatic multithresholding to perform both dark and light images of the eye to identify tumor-like region. Thresholding is a crucial method for segmenting images. In comparison to a gray-level image with 256 levels, the segmented image produced by thresholding has the advantages of smaller storage volume, quick processing, and ease of manipulation. This has made thresholding techniques quite popular in recent years. A successful segmentation will distinguish between pixels with similar values to improve contrast and separate objects from the background. In many image processing applications, image regions are anticipated to have uniform properties (such as hue or gray level), indicating that they are parts of the same object or its facets and suggesting the prospect of effective segmentation. There are two categories of thresholding techniques: bilevel and multilevel. First, get a histogram from the image with the background removed by moving the *x* axis of the histogram. Then, the *y* axis of the histogram, which shows the number of pixels, goes from the highest number, i.e., maximum point to the lowest number, i.e., minimum point. This maximum point (ma) and minimum point (mi) show a smooth status; on clearer region of the tumor cells, its histogram is quickly going down. From the falling curve (Figure 2), we can figure out the smooth rate; the smooth rate can be expressed in

(1) $$\begin{array}{c} \text{SR}=\frac{\sqrt[{2}]{\sum_{j=\text{ma}}^{\text{mi}}\left(\left(j,1\right)-\left(j+1,1\right)\right)}}{\text{ma}-\text{mi}}. \end{array}$$

If the curves in the histogram gradually decrease in slope from its maximum point to its minimum point, this indicates that the image is dark and that its smooth rate is high. It indicates that the sharpness is low and that there are many dark pixels in the image. If the curve in the histogram drops off suddenly from its maximum point to its minimum point, this indicates that the image is bright and that its smooth rate is low. It indicates that there is a higher contrast, as well as a high quantity of pixels that are bright. When we reach a steady rate, the value of the threshold for the subsequent stage will be calculated on its own automatically. The histogram of each division is utilized to calculate thresholds, and each pixel's grayscale value is compared to the threshold to classify it. When image *g*(*a*, *b*) classes employ threshold *t*, it can be expressed as

(2) $$\begin{array}{c} g\left(a,b\right)=\left\{\begin{array}{c} 1\text{ if }g\left(a,b\right)\text{ greater than threshold value},\\ \;0\text{ if }g\left(a,b\right)\text{ greater than or equal to threshold value}. \end{array}\right.\; \end{array}$$

Multithresholding gathers similar data based on the features in a single group of clusters and dissimilar ones in separate clusters. The following steps shows the steps of automatic multithresholding:

1. Apply Otsu multithresholding technique and get a threshold value (*G*1, *G*2)
2. Apply Otsu multithresholding algorithm to separate *G*1 into two groups (*G*1a, *G*1b) and *G*2 into two groups (*G*2a, *G*2b) (*G*2a, *G*2b)
3. Third, apply Otsu multithresholding method to divide *G*1a, *G*1b, *G*2a, and *G*2b into *G*1a+, *G*1a, *G*1b+, *G*1b, *G*2a+, *G*2a, *G*2b+, and *G*2b

Automatic multithresholding method groups a tumor-like region (TLR) into a single cluster [10]. Once the TLR is identified (Figure 3), the cancerous cell and noncancerous cells are needed to be differentiated, because not all the tumors lead to retinoblastoma. The next step is to classify the retinoblastomic cell and nonretinoblastomic cell; this classification is carried out using AlexNet and ResNet50 algorithms.

### 3.1. ResNet50

An existing deep learning framework for classifying photos is called ResNet50. It is based on the convolutional neural network (CNN, or Conv Net), a deep neural network type typically employed for image analysis. A million photos from a thousand different categories were used to train ResNet50, which contains 50 layers. A convolution block and an identity block are included in each of the ResNet50 model's five stages. Each identity block has the same amount of identity blocks, and each convolution block has three levels of convolution. Additionally, the model has more than 23 million trainable parameters, demonstrating its deep architecture and ability to recognize images more accurately.

Residual networks are made up of several successive residual modules, which are ResNet's basic building blocks [11]. As the network learns deeper, it gets harder to train people. In most cases, the input feature map is followed by a convolutional filter, a nonlinear activation function, and a pooling operation. The next layer is then the output. This is where the back propagation algorithm is put into action. As the network gets bigger, it gets harder and harder to bring everything together. ResNet50 is built in four stages. The size of the image when it comes in is 224 × 224 × 3. Every ResNet structure does the first convolution and max pooling differently, using kernel sizes of 7 × 7 and 3 × 3, respectively. Next, the first stage of the network begins. It is made up of 3 residual blocks, each of which has 3 layers. The kernels used to do the convolution operation with all three layers of the first stage block are 64, 64, and 128 bits in size, respectively. The wavy arrows show that the relationship is clear. The dashed arrow shows that the process of bending in the residual block is done with stride 2. This means that the height and width of the input will be cut in half, but the width of the channel will be doubled. As we move from one moment to the next, the width of the channel is doubled and the length of the input is cut in half. Constriction pattern is used for large networks like ResNet50 and ResNet152. For every extra process *F*, three layers are moved on top of each other. The three layers are made up of 1 × 1, 3 × 3, and 1 × 1 convolution. The 1 × 1 convolution layers are in charge of making the dimensions smaller and then changing them. With less input and output dimensions, the 3 × 3 layer is still a bottleneck. Lastly, the network has an average pooling layer followed by a layer with 1000 neurons that are connected to each other [12].

### 3.2. AlexNet

AlexNet [13] outperformed conventional deep learning algorithms. It was a revolution in deep learning for visual recognition and classification. The first convolutional layer uses 96 11 × 11 receptive filters, with normalization of local response (LRN). With a 2-step stride, 3 × 3 filters are used in max pooling. Five-by-five filters are employed in the second layer. Three-by-three filters with 384, 384, and 296 feature maps are used in the third, fourth, and fifth convolutional layers. Following are two FC dropout layers, followed by a Softmax layer. This approach uses the same number of feature maps to train two networks that are identical. Dropout and LRN are introduced by this network. LRN can be applied to single channels or to feature maps, which normalize a *N* × *N* patch depending on neighborhood values. Second, LRN functions across feature maps or channels.

Figure 4 illustrates the architecture of the proposed methodology where the input image is given into autothresholding method to identify the tumor-like region (TLR). The TLR is identified by using the OTSU autothresholding method, where it applies clustering technique to group the similar set of images based on equations (1) and (2). In this work, the performance of the two variants of convolutional neural network (CNN) algorithms, ResNet and AlexNet, is compared. Automated thresholding method identifies TLR but not all the tumors are malignant.

Tumors that are cancerous or malignant have the potential to metastasize to adjacent tissue, glands, and other body organs. Metastases are the new tumors (mets). After treatment, cancerous tumors may return (cancer recurrence). It may be fatal to have these tumors.

- Nonmalignant: benign tumors are rarely life-threatening and are not cancerous. They are localized, which means that they frequently do not spread to other areas of the body or impact neighboring tissue. Treatment is not necessary for many benign tumors. On the other hand, certain benign tumors press against other bodily parts and require medical attention
- Precancerous: if left untreated, these noncancerous tumors may develop into malignancy. The CNN variants are used to identify the cancerous region and classify the images

## 4. Dataset and Implementation

MathWorks [14] is the source of our dataset, which aims to construct a model for detecting degenerative disease (DR). The MRI, CT, and fundus procedures are utilized to examine the eyeballs. MRI images demonstrate the ligamentous engagement in the extraocular extension highlighted in this scan. Retinoblastoma might show up as both hyper- and hyporeflective on an MRI scan. The calcified area is obvious on the CT image, and the eye is nucleated by the huge tumor. Patients' fundus images are captured using the Retcam pediatric camera. Patients between the ages of 12 and 20 are targeted for this study. According to Table 1 and Figure 5, the dataset contains high-resolution eye pictures that have been rated by skilled specialists into five classes (I-V). Each picture is rated on a scale of I to V, where I represents no retinoblastoma, II represents weak retinoblastoma, III represents substantial retinoblastoma, IV represents extreme retinoblastoma, and V represents proliferating retinoblastoma. In the proposed implementation, 128 patches are created for each of the 1024 × 1024 pixel input images. The data from each patch is then further reformed: they are turned counterclockwise by 90, 180, 270, and 360 degrees, and each one is inverted horizontally afterward. In this way, eight alternative patches are generated for each source patches, resulting in 1024 training parameters for the proposed system performance analysis. A total of 183,747 trainable parameters are built using the dataset for performance analysis.

The proposed methodology was implemented in a system with a configuration of i7 11th generation GPU and 16 GB of RAM. Programming language used for the implementation is Python 3.10.5 with Keras and TensorFlow as the backend structure. From the dataset (278), 70% (194) of the image set is utilized for training and 30% (84) of the dataset is used for testing. The number of epochs attempted in this implementation is 10 which was sufficient for the performance converge. The ReLU and Softmax optimizer are used as the activation function and the assumed learning rate is 0.0001.

## 5. Results and Discussion

A retinoblastoma model is proposed, and its performance is evaluated using metrics including accuracy, precision, recall, and *F*1 score. To demonstrate the effectiveness of the suggested algorithm, the existing techniques XGBoost, random forest, CNN, and KNN are compared with RB-AlexNet and RB-ResNet.

The performance metrics is analyzed using the following equations:

(3) $$\begin{array}{c} \text{Accuracy}=\frac{\text{TP}+\text{TN}}{\text{TP}+\text{TN}+\text{FP}+\text{FN}},\\ \text{Precision}=\frac{\text{TP}}{\text{TP}+\text{FP}},\\ \text{Recall}=\frac{\text{TP}}{\text{TP}+\text{FN}},\\ F1\text{ score}=2*\frac{\text{Precision}*\text{recall}}{\text{Precision}+\text{recall}}. \end{array}$$

The ResNet50 result includes the following: from a total of 278 images, 258 images are true positives (TP), i.e., correctly classified RB images; 11 images are false positives (FP), i.e., incorrectly classified as RB images; 8 images are false negative (FN), i.e., incorrectly classified as normal images; and 1 image is true negative (TN), i.e., correctly classified as normal image. The AlexNet result includes the following: from a total of 278 images, 243 images are TP, 18 images are FP, 15 images are FN, and 2 images are TN.  Figure 6 depicts the confusion matrix for the proposed algorithm with ResNet50 and AlexNet architecture. An analysis of the confusion matrix for a convolutional neural network (CNN) reveals which classes the model predicts properly and which classes it predicts poorly. The “evaluate” function can be used to gauge the performance of a convolutional neural network. The test results are used as the method's parameters. The data is first visualized on the console with the help of the “matplotlib” library and “imshow” methods.

Figure 7 shows the classified images with and without retinoblastoma using the proposed CNN models.  Table 2 describes the overall performance of the proposed CNN model with reference to assumed performance metrics. The ResNet50 architecture obtained the highest accuracy of 93.16 among all other models. From the simulated metrics, it is evident that the ResNet50 model is superior to all other existing models in terms of accuracy, precision, recall, and *F*1 score.

## 6. Conclusion

Diabetes-related retinoblastoma is a serious cause of vision loss. Retinoblastoma lesions have a significant clinical impact if they can be accurately diagnosed. Early diagnosis and treatment are essential since early discovery can successfully prevent vision loss. Diabetic retinopathy diagnosis can be improved by using retinoblastoma automated categorization of fundus pictures, which can benefit clinicians. In order to categorize retinoblastoma fundus pictures and automate multithresholding learning for feature extraction from fundus photos, specifically convolutional neural networks for detecting retinoblastoma are described in this research. In this paper, the CNN-based multithresholding technique is investigated on the Retinoblastoma 2022 dataset. The implementation is based on the AlexNet and ResNet50 backbone designs. The highest empirical classification performance is ResNet50 with 93.16 percent, and our results show that retinoblastoma prediction and classification are more accurate than other existing models.

## Figures and Tables

**Figure 1:** Fundus images of patients with and without RB.

**Figure 2:** Histogram representation for RB image.

**Figure 3:** RB image with TLR.

**Figure 4:** Architecture of the proposed methodology.

**Figure 5:** Different stages of retinoblastoma.

**Figure 6:** Confusion matrix for CNN models.

**Figure 7:** Classified images with and without RB.

**Algorithm 1:** 

**Table 1:** Classes of retinoblastoma.

Category	Degree	Number
I	No RB	35
II	Weak RB	64
III	Substantial RB	74
IV	Extreme RB	68
V	Proliferate RB	37

**Table 2:** Performance comparison of the proposed vs. existing models.

Framework	Accuracy	Precision	Recall	*F*1 score
XGBoost [6]	82	87	86	86
Random forest [6]	85	90	89	88
KNN [6]	84	88	89	88
CNN [7]	87	92	93	92
AlexNet	88.12	93.10	94.18	93.64
ResNet50	93.16	95.91	96.99	96.44

## Data Availability

The data shall be made available on request from the corresponding author.
